# The Roles of circMTO1 in Cancer

**DOI:** 10.3389/fcell.2021.656258

**Published:** 2021-06-30

**Authors:** Wei Liu, Yuanyuan Xiong, Renhua Wan, Renfeng Shan, Jianfeng Li, Wu Wen

**Affiliations:** Department of General Surgery, The First Affiliated Hospital of Nanchang University, Nanchang, China

**Keywords:** circular RNAs, circMTO1, cancers, microRNA, tumor progression

## Abstract

Circular RNAs (circRNAs) are a recently discovered type of covalently-closed circular non-coding RNAs, mainly formed by non-sequential back-splicing of precursor mRNAs (pre-mRNAs). Recent studies have demonstrated that circRNAs can have either oncogenic or tumor-suppressor roles depending on the cellular context. CircRNA mitochondrial tRNA translation optimization 1 (circMTO1), a recently reported circular RNA originating from exons of MTO1 located on chromosome 6q13, was proved to be abnormally expressed in many malignant tumors, such as hepatocellular carcinoma, gastric carcinoma and colorectal cancer, resulting in tumor initiation and progression. However, there are no reviews focusing on the roles of circMTO1 in cancer. Here, we first summarize the main biological characteristics of circMTO1, and then focus on its biological functions and the possible underlying molecular mechanisms. Finally, we summarize the roles of circMTO1 in cancer and discuss future prospects in this area of research.

## Introduction

Circular RNAs (circRNAs), which represent a special type of endogenous non-coding RNAs, have attracted great attention in the RNA field in recent years. Unlike linear RNAs, which have terminal 5′ caps and 3′ tails, circular RNAs are covalently closed loops without polyadenylated tails or 5′–3′ polarity (Chen and Yang, 2015; Qu et al., 2015). CircRNAs were first identified in RNA viruses in the 1970s (Sanger et al., 1976). Unfortunately, circRNAs were only serendipitously reported following this discovery, and were typically considered to be products of intermediates of intron lariat debranching or RNA splicing errors. Thus, circRNAs were largely ignored and were considered unlikely to play a critical role in biological processes (Jeck et al., 2013). However, with the emergence of bioinformatics and RNA deep sequencing technology, recent studies found abundant circRNAs of different types in mammalian cells. Moreover, circRNAs appear to be a conserved and diverse class of stable RNA molecules (Jeck et al., 2013; Memczak et al., 2013; Salzman et al., 2013; Zhang et al., 2013; Guo et al., 2014; Li Y. et al., 2015; Li Z. et al., 2015). Thousands of circRNAs have been detected in human tissues by high-throughput sequencing, and they are now known to be widely expressed in eukaryotic cells (Xia et al., 2017). In some cases, the expression level of a circRNA can be 10-fold higher than that of its cognate linear mRNA (Jeck et al., 2013). Generally, circRNAs are primarily located in the cytoplasm, and only a small number of circRNAs reside in the nucleus (Memczak et al., 2013). Approximately one third of all circRNA molecules appear to be conserved among different species (Xia et al., 2017), with dynamic tissue-specific expression changes at different developmental stages (Salzman et al., 2013). Notably, circRNAs exhibit longer half-lives than mRNAs, and can serve as important regulators of transcription and post-transcriptional gene expression (Chen et al., 2016).

According to the positions of their encoding genes, circRNAs can be categorized as exonic circRNAs (ecircRNAs) (Jeck et al., 2013), intronic circRNAs (ciRNAs) (Aucamp et al., 2016), and exon-intron circRNAs (EIciRNAs) (Li Z. et al., 2015). Generally, most ecircRNAs are cytoplasmic (Jeck et al., 2013; Memczak et al., 2013), while ciRNAs and EIciRNAs are mainly found in the nucleus, indicating that they have a potential role in transcriptional regulation (Li Z. et al., 2015; Chen et al., 2016). In contrast with the canonical splicing of linear RNAs most circRNAs discovered today are produced by back-splicing of pre-mRNAs, which (Chen, 2016; Chen et al., 2017). Jeck et al. (2013) proposed two models for the biogenesis of circRNAs, respectively, named intron-pairing-driven circularization and lariat-driven circularization. Shortly thereafter, another model of circRNA biogenesis was also reported. This model assumes that flanking introns are connected via RNA binding proteins (RBPs), bringing the splice donor and acceptor closer to each other, thereby facilitating the circularization of exons (Figure 1; Ashwal-Fluss et al., 2014; Conn et al., 2015). In addition, using advanced high-throughput sequencing and bioinformatics analysis, the roles of circRNAs were clarified (Han et al., 2018). Their functions in gene regulation are as follows:

**FIGURE 1:** The biogenesis of circular RNAs (circRNAs). **(A)** Lariat-driven circularization. EIciRNAs or ecircRNAs are generated by exon skipping. The 3′splice site is attacked by exons 5′, forming an mRNA composing of exon 1 and exon 4 and an RNA lariat embodying skipped exon 2 and exon 3. Then, an RNA double lariat and an EIciRNA were further generated. **(B)** Intron-pairing-driven circularization. The pairing of the inverted complementary sequences in the flanking introns makes the splicing sites close to each other, promoting the circularization of intervening exons. And EIciRNAs or ecircRNAs are formed by retaining or removing introns. **(C)** RNA-binding protein (RBP)-driven circularization. RBPs binding to the flanking introns, which act as a bridge to make flanking introns close to each other, facilitating the process of circularization.

(1) Regulating transcription or alternative splicing. RNA can be bound by stable nuclear circRNAs, thereby promoting transcription. For example, EIciRNAs can undergo a specific RNA-RNA interaction with U1snRNPs (U1 small nuclear ribonucleoproteins), and the resulting complexes can interact with the RNA Pol II transcription complex to enhance gene expression (Li Z. et al., 2015). Moreover, circRNAs can reduce linear mRNA production by competing with canonical pre-mRNA splicing to alter the composition of processed mRNAs (Chen et al., 2017).
(2) Acting as competing endogenous RNAs (ceRNAs) or sponging microRNA (miRNAs). CircRNAs contain miRNA response elements (MREs), and therefore might act as ceRNAs to reduce miRNA binding to their target genes, thereby indirectly regulating the expression of the miRNA targets (Hansen et al., 2013; Hou and Zhang, 2017). For example, circMTO1 was found to inhibit the initiation and development of gastric carcinoma by increasing the expression of Phosphatidylethanolamine-binding protein 1 (PEBP1) via sponging of miR-3200-5p (Hu et al., 2020).
(3) Protein translation. Increasing numbers of studies show that circRNAs have protein-coding potential (Jeck and Sharpless, 2014; Legnini et al., 2017). It was found that one way to achieve translation of circRNAs is driven by an internal ribosome entry sequence (IRES) to promote direct binding of the ribosome or initiation factors to the translatable circRNA (Lener et al., 2015; Legnini et al., 2017; Pamudurti et al., 2017; Zhang et al., 2018).
(4) Interaction with RBPs. CircRNAs may regulate the transcription of target genes through protein binding, and enhancing protein-protein interactions (Chen et al., 2017). For example, there is direct binding between Y-box binding protein-1 (YBX1) and circFAT1 (e2) from exon 2 of FAT atypical cadherin 1 (FAT1), which can inhibit the progression of gastric cancer (Fang et al., 2019).

In recent years, circRNAs have garnered great interest in the RNA field due to their critical roles in human disease initiation and progression, especially in tumorigenesis (Guarnerio et al., 2016; Holdt et al., 2016; Bai et al., 2018; Geng et al., 2018; Luan et al., 2018; Zhou et al., 2018; Guo et al., 2019). Undoubtedly, expanding our understanding of the roles circRNAs play in the stemness, drug resistance, and potential biomarkers of cancer will provide new insights for tumor therapy (Lux and Bullinger, 2018; Qu et al., 2018; Su et al., 2019). The circRNA mitochondrial tRNA translation optimization 1 (circMTO1) has been verified to play a critical regulatory role in tumor progression by sponging multiple miRNAs, including miR-6893 and miR-9 (Han et al., 2017; Chen M. et al., 2019). Moreover, circMTO1 was found to promote tumorigenesis in cervical cancer cells by sponging miR-6893 (Chen M. et al., 2019). However, circMTO1 was also found to suppress hepatocellular cancer growth by sponging miR-9 to up-regulate p21 expression (Han et al., 2017). This indicates that circMTO1 plays dual roles in tumor progression by sponging different miRNAs and affecting different target proteins or signaling pathways. Considering the importance of circMTO1 in the field of non-coding RNAs and the underlying mechanisms of its roles in tumor development, summarizing the published data will help further research in this respect. In the subsequent sections, we will summarize the current researches on the clinical significance of circMTO1 in the initiation and progression of human tumors and the underlying mechanisms, with the aim to inspire new directions for the clinical diagnosis and targeted therapy of tumors.

## The Biological Features of circMTO1

The circular RNA MTO1 (circMTO1) originates from exons 2 and 3 of the mitochondrial tRNA translation optimization 1 (MTO1) gene with a 318bp splice length (Figure 2), and was first reported in hepatocellular carcinoma (Han et al., 2017; Fan et al., 2019). CircMTO1 is formed by non-linear splicing of the MTO1 pre-mRNA, but it remains unclear whether circMTO1 influences the transcript levels of the linear mRNA (Li K. et al., 2020). Thus, the relationship between circMTO1 and linear MTO1 needs further research. Similar to other circRNAs, circMTO1 is a single chain circular RNA without a polyadenylated tail or 5′–3′ polarity (Barrett and Salzman, 2016; Rao et al., 2018). The closed structure makes circMTO1 more resistant RNA degradation. It has been demonstrated that circMTO1 is abundantly and stably expressed in different human tissues, where it is mainly present in the cytoplasm (Li Z. et al., 2019; Wang et al., 2019; Hu et al., 2020). Receiver operating characteristic curve analysis indicated that serum circMTO1 may act as a potential diagnostic biomarker for liver fibrosis in chronic hepatitis B (CHB) patients. Overexpression of circMTO1 was found to suppress the activation of hepatic stellate cells (HSCs) by transforming growth factor-β1, thereby inhibiting the progression of liver fibrosis (Wang et al., 2019). Moreover, overexpression of circMTO1 was found to attenuate acute kidney injury (AKI) by sponging miR-337 and regulating the expression of Kruppel like factor 6 (KLF6) (Shi et al., 2020). In addition, circMTO1 was also confirmed to be involved in the initiation and development of various tumors (Zhang X. et al., 2019; Wang X. et al., 2020).

**FIGURE 2:** Genomic locus of MTO1 and circMTO1. In humans, MTO1 gene is located on chromosome 6 at chr6q13 (73461737–73509236), gene ID: 25821, and contains 14 exons (www.ncbi.nlm.nih.gov/gene/25821). The exons that generate circMTO1 are located at chr6q13 (74175931–74176329).

## circMTO1 Functions as a miRNA Sponge

The available data on circMTO1 from PubMed and other relevant databases indicates that circMTO1 can act as a miRNA sponge to regulate gene expression by interacting with several miRNAs (Figure 3), most of which have oncogenic roles, such as miR-19b-3p and miR-630, which promote tumor cell proliferation in rectal cancer and osteosarcoma, respectively. By sponging miR-19b-3p and miR-630, circMTO1 inhibits their activity and thus suppress the growth of cancer cells (Fan et al., 2019; Liu et al., 2021). However, circMTO1 sponges miR-6893 to promote the proliferation, migration, invasion of cervical cancer cells (Chen M. et al., 2019). CircMTO1 is also able to sponge miR-3200-5p and miR-17 in gastric carcinoma and lung adenocarcinoma, respectively (Zhang B. et al., 2019; Hu et al., 2020). In addition, circMTO1 also plays a role in the in the progression of ovarian cancer by regulating miR-760 and miR-182-5p (Li L. et al., 2020; Wang N. et al., 2020). MiR-9 is a target of circMTO1 in hepatocellular carcinoma and renal cell carcinoma (Han et al., 2017; Li K. et al., 2020). In glioblastoma, there is a potential binding site for circMTO1 sponging of miR-92, through which it regulates cancer progression (Zhang X. et al., 2019). On the other hand, circMTO1 negatively regulates miR-17-5p expression, and it was found to be related to the progression of prostate cancer, including the pathological T stage and N stage (Hu and Guo, 2020). Table 1 shows the miRNAs regulated by circMTO1 in various tumors.

**FIGURE 3:** Schematic diagram of circMTO1 function as a miRNA sponge. CircMTO1 exits the nucleus and can act as a sponge for the designated miRNAs, which regulate their respective target genes, thereby promoting or inhibiting tumor progression. T-shaped arrow: inhibition; Standard-shaped arrow: stimulation.

**TABLE 1:** Expression levels and functions of circMTO1 in different tumors.

Tumor type	Expression level	Target miRNAs	Target proteins	Associated cellular process	Clinicopathological features	References
Cervical cancer	UP	miR-6893	S100A1; Beclin1; p62	Promotes cell proliferation, migration, invasion, and inhibits apoptosis	−	Chen M. et al., 2019
Gallbladder cancer	UP	−	−	−	TNM stage, lymph node metastasis, distant metastasis, poorer progression-free survival, poorer overall survival,	Wang X. et al., 2020
Rectal cancer	Down	miR-19b-3p	JAK1/STAT3; AMPK	Inhibits cell proliferation, migration, invasion, and induces apoptosis	−	Fan et al., 2019
Osteosarcoma	Down	miR-630	KLF6	Inhibits cell proliferation, migration, invasion, and induces apoptosis	Enneking stage, poorer overall survival	Liu et al., 2021
Glioblastoma	Down	miR-92, miR-630	WWOX	Inhibits cell proliferation, induces apoptosis	Advanced clinical stage, poorer overall survival	Rao et al., 2018; Zhang X. et al., 2019
Gastric carcinoma	Down	miR-3200-5p, miR-199a-3p	PEBP1; PAWR	Inhibits cell proliferation, migration, invasion, and induces apoptosis	Higher TNM stage, poorer overall survival	Hu et al., 2020; Song et al., 2020
Lung adenocarcinoma	Down	miR-17	QKI-5	Inhibits cell proliferation	Lymph node metastasis, advanced clinical stage, poorer overall survival, poorer progression-free survival	Zhang B. et al., 2019
Ovarian cancer	Down	miR-760, miR-182-5p	SOCS3; KLF15	Inhibits cell proliferation, migration, invasion	Poorer overall survival	Li L. et al., 2020; Wang N. et al., 2020
Hepatocellular carcinoma	Down	miR-9, miR-9-5p	p21; NOX4	Inhibits cell proliferation, migration, invasion, and induces apoptosis	Poorer overall survival	Han et al., 2017; Wang J. et al., 2020
Renal cell carcinoma	Down	miR9 miR223	LMX1A	Inhibits cell proliferation, migration, invasion	Poorer overall survival	Li K. et al., 2020
Prostate cancer	Down	miR-17-5p	−	Inhibits cell proliferation and invasion	Pathological T/N stage, poorer overall survival, poorer disease-free survival	Hu and Guo, 2020
Bladder cancer	Down	miR-221	E-cadherin/N-cadherin	Inhibits migration, invasion	Distant metastasis, poorer overall survival, poorer disease-free survival	Li Y. et al., 2019
Colorectal cancer	Down	−	Wnt/β-catenin	Inhibits cell proliferation and invasion	TNM stage, lymph node metastasis, poorer overall survival	Ge et al., 2018
Breast cancer	Down	−	TRAF4; Eg5	Inhibits cell proliferation	Poorer overall survival	Liu et al., 2018

## circMTO1 in Various Human Cancers

Recent studies have reported that circRNAs has both oncogenic and tumor-suppressive roles depending on the cellular context. With advancement of circRNA research, differences in circMTO1 expression have been detected in normal and diseased tissue. Many studies have verified that circMTO1 is abnormally expressed in a large number of tumors, including rectal cancer, osteosarcoma, glioblastoma, cervical cancer, gallbladder cancer, gastric carcinoma, lung adenocarcinoma, ovarian cancer, hepatocellular carcinoma, renal cell carcinoma, prostate cancer, bladder cancer, colorectal cancer, and breast cancer (Han et al., 2017; Liu et al., 2018; Rao et al., 2018; Chen M. et al., 2019; Fan et al., 2019; Li Y. et al., 2019; Zhang B. et al., 2019; Hu and Guo, 2020; Hu et al., 2020; Li K. et al., 2020; Li L. et al., 2020; Liu et al., 2021; Song et al., 2020; Wang J. et al., 2020; Wang N. et al., 2020; Wang X. et al., 2020). Furthermore, upregulation of circMTO1 expression was reported to inhibit cell proliferation in rectal cancer, osteosarcoma, glioblastoma, gastric carcinoma, lung adenocarcinoma, ovarian cancer, renal cell carcinoma, hepatocellular carcinoma, prostate cancer, colorectal cancer, and breast cancer. Moreover, overexpression of circMTO1 was also found to suppress cell migration and invasion in rectal cancer, osteosarcoma, renal cell carcinoma, gastric carcinoma, ovarian cancer, hepatocellular carcinoma, and bladder cancer. Downregulation of circMTO1 expression showed a positive correlation with lymph-node metastasis in lung adenocarcinoma and colorectal cancer, while low expression of circMTO1 was closely related to poorer overall survival in glioblastoma, lung adenocarcinoma, hepatocellular carcinoma, prostate cancer, bladder cancer, and colorectal cancer. These studies show that the expression of circMTO1 is dynamically regulated during tumor progression, and that circMTO1 exerts its regulatory functions through multiple ways.

### Cervical Cancer

Globally, cervical cancer is the fourth most common cancer affecting women. In spite of significant improvements in the treatment of cervical cancer due to the introduction of angiogenesis inhibitors, the 5-year overall survival rate is still low (Kagabu et al., 2019). It is therefore essential to reveal the molecular mechanisms driving the development and progression of cervical cancer, which may provide useful novel therapeutic targets.

In 2019, it was found that circMTO1 is significantly upregulated in cervical cancer tissues and cell lines. CircMTO1 interacts directly with miR-6893, which was found to restore the chemoresistance of cervical cancer cells. In addition, they found that S100 calcium binding protein A1 (S100A1) is a downstream target through which circMTO1/miR-6893 promotes the cell proliferation, migration and invasion of cervical cancer. Moreover, western blot analysis revealed that circMTO1 and miR-6893 inhibitors promote Beclin1 expression and downregulated p62 levels, thereby inhibiting apoptosis. Additionally, the autophagy inhibitor 3-MA increased the apoptosis rate of HeLa cells treated with circMTO1 and miR-6893 inhibitors (Chen M. et al., 2019). These results suggested that circMTO1 might play a critical role in cervical cancer development, which makes it a potential new therapeutic target for cervical carcinoma.

### Gallbladder Cancer

Although gallbladder cancer (GBC) is a rare disease overall, it is the most frequent malignant tumor of the biliary tract worldwide, as well as having higher mortality than in many other types of cancer (Kanthan et al., 2015). Moreover, most patients are diagnosed too late and thus have a poor prognosis. Even where surgical resection is possible, the prognosis of GBC is still unsatisfactory (Dwivedi et al., 2015; Wang S. et al., 2020). Hence, it is urgent to discover effective early biomarkers and therapeutic targets.

Wang X. et al. (2020) reported that circMTO1 expression was significantly upregulated in GBC tumor tissues and the increase was detectable in the plasma. The expression of circMTO1 was found to be closely correlated with lymph node metastasis, TNM stage, tumor size, differentiation, and distant metastasis. Overexpression of circMTO1 acted as an independent prognostic factor of shorter progression-free survival and overall survival in GBC patients. Furthermore, the increase of plasma circMTO1 levels was significantly related to tumor development (Wang X. et al., 2020). These results demonstrated that circMTO1 might act as a potential early diagnostic and therapeutic biomarker for GBC.

### Rectal Cancer

Rectal cancer is a malignant tumor with a high mortality rate due to its strong invasion and metastasis ability, as well as a high recurrence rate (Wietek and Kratt, 2012; Yang et al., 2015). Although various treatment methods such as minimally invasive and laparoscopic surgery have made great advances, the prognosis of rectal cancer patients remains poor (Fleshman et al., 2019). Accordingly, it is urgent to discover novel efficient treatment methods for rectal cancer.

Fan et al. (2019) demonstrated that circMTO1 expression was significantly reduced in rectal cancer tissues compared with adjacent normal tissue specimens. They also found that overexpression of circMTO1 could inhibit cell proliferation, migration and invasion while promoting apoptosis by downregulating miR-19b-3p. Moreover, overexpression of circMTO1 exerted an antitumor effect by negatively regulating miR-19b-3p to suppress the Janus kinase 1 (JAK1)/signal transducer and activator of transcription 3 (STAT3) and AMP-activated protein kinase (AMPK) signaling pathways, inhibiting SNU-61 and SW837 cell proliferation, migration, and invasion and promoting apoptosis (Fan et al., 2019). These results indicated that circMTO1 might have an inhibitory effect on rectal cancer, which makes it a potential therapeutic target and prognostic biomarker.

### Osteosarcoma

Osteosarcoma is an invasive and most prevalent type of primary bone malignancy that derives from osteogenic mesenchymal cells (Misaghi et al., 2018). Despite significant advancements in recent decades, the prognosis of osteosarcoma patients is not satisfactory (Marina et al., 2004; Harrison et al., 2018). Hence, there is an urgent need to investigate the underlying mechanisms of osteosarcoma progression and explore novel therapeutic targets.

Liu et al. (2021) verified that lower level of circMTO1 was expressed in osteosarcoma tissues and cell lines. Moreover, low expression level of circMTO1 was associated with Enneking stage and poor overall survival. Overexpression of circMTO1 restrained cell proliferation, migration and invasion, promoted apoptosis in HOS and U2OS cells. Furthermore, they also confirmed that overexpression of circMTO1 could promote Kruppel like factor 6 (KLF6) expression by sponging miR-630, thereby playing a tumor suppressor role in osteosarcoma (Liu et al., 2021). In summary, these findings suggest that circMTO1 may be a novel therapeutic target for osteosarcoma.

### Glioblastoma

Glioblastoma is one of the brain tumors with the highest incidence, and is considered an invariably lethal malignancy due to its quick reproduction (Delgado-Lopez and Corrales-Garcia, 2016). At present, the standard treatments for glioblastoma patients under 70 years old mainly relies on surgical resection plus adjuvant temozolomide (TMZ) (Hanif et al., 2017). However, its effects are unsatisfactory because of the chemoresistance of glioblastoma, with very poor overall survival (Linz, 2010). Hence, it is imperative to explore the molecular mechanisms driving the progression of glioblastoma and find novel therapeutic targets.

In recent years, the potential functions of circMTO1 in glioblastoma and underlying molecular mechanisms have been explored. Zhang X. et al. (2019), as well as Rao et al. (2018), reported that circMTO1 expression was significantly downregulated in glioblastoma tissue samples and cell lines. Moreover, circMTO1 expression decreased with the progression of clinical stages, while overexpression of circMTO1 restrained cell proliferation and induced apoptosis. Zhang X. et al. (2019) found that circMTO1 might serve as a ceRNA binding to miR-92 to upregulate WW domain containing oxidoreductase (WWOX) expression and inhibit the proliferation of glioblastoma cells. Moreover, Rao et al. (2018) also found that circMTO1 could attenuate the resistance of glioblastoma cells to TMZ, but its downstream genes have not been further studied. In summary, all these data prove that circMTO1 is involved in glioblastoma pathogenesis and may act as a novel therapeutic target of glioblastoma.

### Gastric Carcinoma

Gastric carcinoma (GC) is the most common gastrointestinal malignancy and a major cause of cancer-related deaths worldwide (Thrift and El-Serag, 2020). Despite a certain amount of progress in recent decades, the 5-year overall survival rate of GC remains low due to the high recurrence rate (Chan et al., 2019). Therefore, it is urgent to study the molecular regulation of GC and discover new biomarkers for early diagnosis, treatment and prognosis of GC.

Hu et al. (2020), as well as Song et al. (2020), reported that the expression level of circMTO1 was much lower in GC tissues. Moreover, low expression of circMTO1 was related to advanced TNM stage, lymphatic invasion, tumor size, and poor overall survival. Overexpression of circMTO1 slowed down GC progression by inhibiting the epithelial-mesenchymal transition (EMT), cell proliferation, migration, and invasion. Hu et al. (2020) reported that circMTO1 had a negative effect on the expression of miR-3200-5p by sponging it. Moreover, circMTO1 was confirmed to compete with phosphatidylethanolamine binding protein 1 (PEBP1) for binding to miR-3200-5p to decelerate the progression of GC (Hu et al., 2020). Furthermore, Song et al. (2020) also found that circMTO1 might serve as a ceRNA that binds to miR-199a-3p, thereby increasing the expression of PRKC apoptosis WT1 Regulator (PAWR), and ultimately effectively inhibiting GC progression. Overall, these findings indicate that circMTO1 exerts a tumor suppressor effect in GC and may be a new therapeutic target for this cancer.

### Lung Adenocarcinoma

Accounting for approximately 40% of all lung cancer cases, lung adenocarcinoma (LUAD) is the most frequent type of lung cancer. Despite major achievements in recent years, the overall survival of most LUAD patients is still poor (Denisenko et al., 2018). Accordingly, it is necessary to more comprehensively understand the molecular mechanisms driving the progression of LUAD to find effective early biomarkers and therapeutic targets.

Zhang B. et al. (2019) found that circMTO1 was downregulated in LUAD tissues compared to normal controls. Moreover, overexpression of circMTO1 could suppress the proliferation of LUAD cells *in vivo* and *in vitro*. Subsequent mechanistic investigations indicated that circMTO1 acts as a sponge for miR-17 to promote the expression of the RNA-binding protein QKI, KH domain containing RNA binding (QKI-5), thereby inhibiting Notch signaling. Furthermore, the increase in QKI-5 expression caused by the overexpression of circMTO1 in turn promoted the expression of circMTO1, further inhibiting the proliferation of LUAD cells (Zhang B. et al., 2019). Overall, these results indicate that circMTO1 plays a negative regulatory role in LUAD and may be a potential prognostic marker and therapeutic target.

### Ovarian Cancer

Ovarian cancer (OVA) is a prevalent and fatal malignancy affecting millions of women worldwide (Khalifa et al., 2019). Although great progress has been made in multiple therapies such as surgery, radiotherapy and chemotherapy, OVA patients still have a poor prognosis, and the 5-year overall survival rate is less than 30% (Prado et al., 2014). Therefore, it is urgent to reveal the molecular mechanisms of OVA carcinogenesis and explore novel therapeutic targets.

Li L. et al. (2020), as well as Wang X. et al. (2020), revealed that circMTO1 expression was downregulated in OVA cell lines. Conversely, upregulation of circMTO1 suppressed the proliferation, migration and invasion of OVA cells. Li L. et al. (2020) found that circMTO1 could absorb miR-760 to promote the expression of suppressor of cytokine signaling 3 (SOCS3), thereby inhibiting the proliferation and migration of OVA cells. In addition, Wang X. et al. (2020) also demonstrated that upregulation of circMTO1 expression could inhibit miR-182-5p to promote Kruppel like factor 15 (KLF15) expression, thereby inhibiting cell proliferation and invasion of OVA cells (Li L. et al., 2020; Wang N. et al., 2020). These results confirmed that circMTO1 plays a critical role in OVA development and may be a new therapeutic target for this highly lethal cancer.

### Hepatocellular Carcinoma

Hepatocellular carcinoma (HCC) ranks among the most commonly diagnosed malignancies and is the third leading cause of cancer-related death. In early stage HCC patients, the optimal approach to surgical hepatic resection can be used for diagnosis and effective treatment, but the prognosis for advanced HCC patients remains unsatisfactory and the overall survival is still poor (Yin et al., 2019). Thus, exploring the molecular biological mechanisms that affect the prognosis of HCC and finding novel prognostic biomarkers is crucial for individualized treatment and better prognosis.

Recent studies have investigated the potential biological function of circMTO1 in HCC and the underlying molecular mechanisms. Han et al. (2017), as well as Wang X. et al. (2020), found that circMTO1 was significantly downregulated in HCC tissues and cell lines. Conversely, overexpression of circMTO1 inhibited the proliferation, migration and invasion of HCC cells, inducing apoptosis. Han et al. (2017) found that circMTO1 could act as a sponge of the oncogenic miR-9 to promote the expression of p21, thereby inhibiting cell proliferation and invasion of HCC cells. In addition, Wang X. et al. (2020) also found that overexpression of circMTO1 could upregulate NADPH oxidase 4 (NOX4) expression by sponging miR-9-5p, thereby promoting apoptosis (Han et al., 2017; Wang J. et al., 2020). Overall, these results suggest that reduced expression of circMTO1 may be a prognostic biomarker, as well as a potential therapeutic target for the treatment of HCC.

### Renal Cell Carcinoma

Renal cell carcinoma (RCC) is by far the most frequent kidney cancer, accounting for approximately 90% of all adult renal malignancies (Siegel et al., 2015). However, the standard method for treating RCC is limited to surgical resection even today. Despite the continuous development of surgical approaches, the prognosis of RCC is still unsatisfactory, with a 5-year overall survival rate of only 5–10% (Garcia and Rini, 2007). Hence, it is of great significance to reveal the underlying mechanisms of RCC progression and find novel therapeutic targets.

In recent years, Li L. et al. (2020) investigated the role of circMTO1 and demonstrated that overexpression of circMTO1 could inhibit the proliferation and metastases in both 786-O and A497 renal cancer cells, while circMTO1 silencing promoted tumorigenesis in OS-RC-2 and SNI2C renal cancer cells. It was found that circMTO1 sponges miR9 and miR223 and thereby reduces their levels. In addition, silencing circMTO1 in RCC could downregulate the miR-9 target LIM homeobox transcription factor 1 alpha (LMX1A), thereby promoting the proliferation and invasion of RCC cells (Li K. et al., 2020). Thus, circMTO1 inhibits the progression of RCC via the circMTO1/miR9/LMX1A axis, suggesting that circMTO1 may be a potential target for RCC therapy.

### Prostate Cancer

Prostate cancer is a leading cancer affecting men, and it remains a major global public health issue (Erratum: Global cancer statistics, 2018). Although great progress has been made in the treatment of prostate cancer, the earl-stage patients who respond well to treatment often suffer from sequelae, even though the survival rates are reasonably high. For advanced patients in which the treatment effect is not satisfactory, the overall survival rate is still poor (Litwin and Tan, 2017). Accordingly, it is necessary to find more biomarkers to help improve the clinical prognosis of prostate cancer.

Hu et al. (2020) corroborated the downregulation of circMTO1 expression in tumor tissues of prostate cancer patients. Moreover, high expression of circMTO1 in tumor tissues was related to a lower pathological T stage and N stages. In addition, circMTO1 was found to inhibit invasion, miR-17-5p expression and proliferation of prostate cancer cells, but the downstream genes need to be further explored (Hu and Guo, 2020). Overall, these results indicate that circMTO1 may be a novel biomarker and therapeutic target for the treatment of prostate cancer.

### Bladder Cancer

Bladder cancer is a common malignancy of the urinary system that is characterized by high morbidity and mortality. Although various advanced therapies have recently become available for bladder cancer patients, the 5-year cancer-specific survival rate remains unsatisfactory (Chen Z. et al., 2019). Therefore, it is of great significance to reveal the molecular mechanisms driving the progression of bladder cancer and explore novel therapeutic targets.

Li Z. et al. (2019) firstly reported that circMTO1 is frequently downregulated in bladder cancer tissues, and the decrease in circMTO1 levels was correlated with increased metastasis and shorter survival of bladder cancer patients. In addition, they also found that circMTO1 could sponge miR-221. Additionally, overexpression of circMTO1 was found to negatively regulate the E-cadherin/N-cadherin pathway by competing for miR-221, thereby inhibiting the epithelial-to-mesenchymal transition (EMT) of bladder cancer cells (Li Y. et al., 2019). Taken together, these results provide comprehensive evidence that circMTO1 is a biomarker for bladder cancer and indicate that circMTO1 may be a new therapeutic target for this highly lethal malignancy.

### Colorectal Cancer

Colorectal cancer (CRC) is one of the most frequent malignancies worldwide. Despite significant progress in diagnosis and treatment, CRC patients with advanced disease still have a poor prognosis (Yuan et al., 2019). Accordingly, it is urgent to clarify the molecular mechanisms that drive the progression of CRC and find more effective therapeutic targets.

Ge et al. (2018) demonstrated that circMTO1 levels were decreased in CRC tissue specimens than in adjacent normal tissues. Moreover, low expression of circMTO1 was related to advanced TNM stage, lymph node metastasis and poor overall survival. Overexpression of circMTO1 inhibited the proliferation and invasion of CRC cells. In addition, further experiments confirmed that circMTO1 suppress the proliferation and invasion of CRC cells by regulating the Wnt/β-catenin signaling pathway (Ge et al., 2018). These results indicate that circMTO1 might be a potential predictor and therapeutic target for CRC.

### Breast Cancer

Breast cancer is a major cause of cancer-associated deaths and the most prevalent malignancy in women (Januskeviciene and Petrikaite, 2019). Most patients are diagnosed too late and have a poor prognosis. Currently, the most commonly used treatment strategy is adjuvant chemotherapy and radiotherapy after surgical resection, but the 5-year overall survival rate of breast cancer still remains low (Castaneda and Strasser, 2017). Hence, it is urgent to discover promising prognostic markers and therapeutic targets for breast cancer.

Liu et al. (2018) demonstrated that monastrol resistance was associated with downregulated circMTO1 expression in breast cancer cells. Conversely, overexpression of circMTO1 reduced the cell viability. In addition, they also found that circMTO1 serves as a ceRNA that binds to tumor necrosis factor receptor associated factor 4 (TRAF4), thereby reducing Eg5 protein levels and reversing monastrol resistance and controlling cell viability (Liu et al., 2018). Thus, circMTO1 may act as a critical functional regulatory factor, and restoration of circMTO1 levels may be a future direction to overcome chemoresistance in breast cancer.

## Conclusion

In this review, we summarized the current research on circMTO1 and highlighted its biological functions and clinical value in a variety of tumors. The expression of circRNAs is cell type- and tissue-specific (Barrett and Salzman, 2016; Qian et al., 2020; Zhang et al., 2020), hinting that circRNAs can have either oncogenic or tumor-suppressor roles, which are influenced by the specific cellular context. Numerous circRNAs are expressed in a tissue dependent manner. Some studies have also shown that the overall levels of circRNA and mRNA are not associated, and the diversity of circular isoforms from specific genes can vary in a group of cell types (Salzman et al., 2013; Szabo et al., 2015). Even in fission yeast, the abundance changes of some circRNAs during nitrogen starvation are independent of their linear isoform (Luo et al., 2018). In summary, these results strongly show that the expression of circRNAs is a dynamically regulated process.

Many studies have demonstrated that circMTO1 acts as a tumor suppressor in most cases, inhibiting the proliferation, migration and invasion of tumor cells, as well as inducing apoptosis. Functionally, circMTO1 was found to serve as a miRNA sponge, competitively binding different miRNAs. CircMTO1 was also found to inhibit multiple signaling pathways such as the AMPK, Wnt/β-catenin, JAK1/STA T3, and E-cadherin/N-cadherin pathways. Moreover, as circRNAs lack polyadenylated tails or 5′–3′ polarity, they are more resistant to exonuclease RNase R digestion and exhibit longer half-lives than linear mRNAs (Barrett and Salzman, 2016). Meantime, some studies found that stable in human body fluids, such as plasma and serum. CircMTO1 was upregulated in plasma samples from GBC patients compared to healthy controls and in human GBC tissues compared to non-tumorous tissues. Its expression levels were closely correlated with lymph node metastasis, TNM stage, tumor size, differentiation, distant metastasis. The area under the receiver operating characteristic curve (AUC) of circMTO1 in plasma was 0.8825 (Wang X. et al., 2020). In another study, circMTO1 was shown to significantly downregulated in serum from chronic hepatitis B (CHB) patients. The low expression level of circMTO1 was negatively associated with liver fibrosis progression. The area under the AUC of circMTO1 in serum was 0.914 (95% CI 0.860–0.953) (Wang et al., 2019), which indicated that liver fibrosis patients from healthy controls could be effectively differentiated by serum circMTO1. Furthermore, circMTO1 was found that other tumor, such as lung adenocarcinoma, bladder cancer and colorectal cancer. The abnormal expression of circMTO1 in tumor tissues is also closely related to clinicopathological features, such as overall survival, lymph node metastasis, distant metastasis, TNM stage and poor prognosis. These properties indicate that circMTO1 might become an ideal diagnostic or prognostic biomarkers in diseases.

CircRNAs are more stable compared with linear RNAs due to their unique structure (Li Y. et al., 2015; Wang et al., 2017), and studies have found that circMTO1 can act as a miRNA sponge to regulate the expression of miRNA and downstream genes (Han et al., 2017; Zhong et al., 2018; Chen M. et al., 2019). These results suggest that circMTO1 can act as a potential therapeutic target. CircMTO1 containing oncogenic miRNAs binding sites can inhibit the proliferation or induce apoptosis of tumor cells. Some strategies might help to achieve more accurate treatment, such as restricting the expression of circMTO1 to certain types of cell through cell specific promoters or designing different therapeutic combinations of circMTO1, miRNAs and/or protein binding sites in the light of sponge maps to target specific carcinogens. Hence, circMTO1 could provide useful information for the clinical diagnosis and treatment.

## Author Contributions

WL wrote the manuscript. YX, RS, WW, JL, and RW coordinated and directed the project. All authors read and approved the manuscript.

## Conflict of Interest

The authors declare that the research was conducted in the absence of any commercial or financial relationships that could be construed as a potential conflict of interest.
